# LATS2 Deletion Attenuates Myocardial Ischemia-Reperfusion Injury by Promoting Mitochondrial Biogenesis

This article has been retracted.

**DOI:** 10.1155/2021/1058872

**Published:** 2021-08-17

**Authors:** Yi Chen, Chen Liu, Jiannan Li, Peng Zhou, Xiaoxiao Zhao, Runzhen Chen, Li Song, Hanjun Zhao, Hongbing Yan

**Affiliations:** ^1^Department of Cardiology, Fuwai Hospital, National Center for Cardiovascular Diseases, Peking Union Medical College, Chinese Academy of Medical Sciences, Beijing, China; ^2^Fuwai Hospital Chinese Academy of Medical Sciences, Shenzhen, China

## Abstract

Reperfusion therapy is the most effective treatment for acute myocardial infarction, but it can damage cardiomyocytes through a mechanism known as myocardial ischemia/reperfusion injury (MIRI). In this study, we investigated whether the large tumor suppressor kinase 2 (LATS2) contributes to the development of myocardial MIRI by disrupting mitochondrial biogenesis. Our *in vitro* data demonstrate that cardiomyocyte viability was reduced and apoptosis was increased in response to hypoxia/reoxygenation (H/R) injury. However, suppression of LATS2 by shRNA sustained cardiomyocyte viability by maintaining mitochondrial function. Compared to H/R-treated control cardiomyocytes, cardiomyocytes transfected with LATS2 shRNA exhibited increased mitochondrial respiration, improved mitochondrial ATP generation, and more stable mitochondrial membrane potential. LATS2 suppression increased cardiomyocyte viability and mitochondrial biogenesis in a manner dependent on PGC1*α*, a key regulator of mitochondrial metabolism. These results identify LATS2 as a new inducer of mitochondrial damage and myocardial MIRI and suggest that approaches targeting LATS2 or mitochondrial biogenesis may be beneficial in the clinical management of cardiac MIRI.

## 1. Introduction

Cardiovascular diseases are the leading cause of death worldwide, especially in developing countries [1]. Acute myocardial infarction (AMI) is a major cause of mortality in cardiovascular diseases. For patients with AMI, a rapid and effective opening of the culprit vessel can rescue ischemic myocardium, reduce infarct size, and improve treatment effects [2, 3]. Reperfusion therapy, including thrombolysis, is the most effective treatment for AMI. However, reperfusion of blood flow brought about by the opening of a culprit vessel can cause damage to cardiomyocytes, known as myocardial ischemia/reperfusion injury (MIRI). Studies have found that about 50% of myocardial necrosis cases are caused by MIRI [4–6]. Therefore, it is important to find out how to attenuate MIRI and improve the efficacy of reperfusion therapy in AMI.

The Hippo signaling pathway uses multiple mechanisms to regulate cell death. For example, cancer cell ferroptosis is induced by the activation of the NF2-YAP pathway [7, 8]. In chemoresistant epithelial ovarian cancer, activation of the TAZ-ANGPTL4-NOX2 axis promotes ferroptotic cell death through ATP depletion [9, 10]. In head and neck squamous cell carcinoma, overexpression of the Hippo/Mst1 pathway contributes to the activation of the *β*-catenin/Drp1 pathway and then mediates mitochondrial death. However, it remains unknown whether the Hippo pathway regulates MIRI-associated cardiomyocyte death.

Recent studies have indicated an association between the Hippo pathway and mitochondrial damage [11–13]. Activation of the Hippo-Yap pathway induces mitochondrial damage through the cGAS/STING/IRF3 signaling, resulting in decreased angiogenesis [14]. Mitophagy, a type of mitochondrial autophagy, is a downstream effector of the Hippo-Yap pathway in gastric cancer cells [15]. Besides, mitochondrial oxidative stress, especially mitochondrial ROS production, is positively managed by the Hippo-Yap pathway in lung fibroblasts [16]. Importantly, the Hippo pathway orchestrates the mitochondrial quality control, especially mitochondrial regeneration and mitochondrial replication in cardiovascular diseases [17]. LATS2 is a novel component of the Hippo pathway. Decreased LATS2 expression has been found to attenuate septic cardiomyopathy through inhibition of the Drp1-related mitochondrial fission. However, overexpression of LATS2 has a cancer-suppressing effect in liver cancer cells by promoting apoptosis [18]. Recent studies suggested a role of LATS2 in regulating cardiomyocyte viability. LATS2 activation or overexpression was associated with a reduced mitochondrial autophagy, resulting in cardiomyocyte apoptosis under an oxidative stress microenvironment. In the present study, we asked whether cardiomyocyte MIRI is under the control of LATS2 and whether the mechanism involves the mitochondrial damage.

## 2. Materials and Methods

### 2.1. Treatment

Cultured H9c2 cardiomyocytes were divided into four groups: (1) control group (CONT), (2) H/R injury group (H/R): hypoxia for 2 h followed by reoxygenation for 2 h, and (3) LATS2 transfection group: cells were infected with LATS2 shRNA adenovirus followed by H/R injury [19, 20].

### 2.2. Cell Viability Assay

H9c2 cardiomyocytes in the logarithmic growth phase were seeded in 96-well plates for 24 h and treated with H/R injury or LATS2 shRNA adenovirus [21]. After incubation for another 24 h, 10 *μ*L of CCK-8 solution was added to cells in each group, and after 2 h, absorbance was measured at 450 nm [22, 23].

### 2.3. Immunofluorescence Apoptosis Assay

Apoptotic cells were visualized using TUNEL staining according to the manufacturer's protocol (Nanjing KeyGen Biotech Co., Ltd.) [24]. Briefly, cells that were cultured on coverslips were fixed using 4% neutral buffered formalin solution at room temperature for 30 min and incubated with 0.3% Triton X-100 at room temperature for 5 min. Subsequently, each sample was supplemented with 50 *μ*L of TUNEL detection reagent for 60 min at 37°C in the dark. The cell nuclei were stained with 5 *μ*g/mL DAPI at 37°C in the dark for 5 min [25]. After adding antifade solution, cells were mounted on slides using glass coverslips. All samples were imaged in three random fields using a fluorescence microscope (magnification, ×100).

### 2.4. Lactated Dehydrogenase (LDH) and Creatine Kinase-MB (CK-MB) Activity Assays

Cell culture supernatants were collected by centrifugation at 1,000 rpm for 10 min [26]. After centrifugation, 100 *μ*L/well supernatant was added to 96-well plates to determine the activities of CK-MB and LDH in each group according to the kit's instructions [27].

### 2.5. Western Blot Assay

Proteins were extracted with RIPA buffer, and protein concentration was determined using a Rapid Gold BCA Protein Assay Kit (Thermo Fisher Scientific). A total of 30 *μ*g protein was separated by 10% sodium dodecyl sulphate-polyacrylamide gel electrophoresis and transferred to polyvinylidene fluoride membranes [28]. After blocking, the membranes were incubated overnight at 4°C with primary antibodies Bax (1 : 1,500; Sigma Aldrich, San Luis, MO, USA), Bcl-2 (1 : 1,500, Sigma Aldrich), and *β*-actin (1 : 2,000, Sigma Aldrich), followed by 1 h incubation with horseradish peroxidase-conjugated secondary antibody (1 : 5,000; Sigma Aldrich). The bands were visualized using an ECL detection kit (Thermo Fisher Scientific) and observed under a Gel-Pro Analyzer version 4.0 (Media Cybernetics, Silver Spring, MD, USA) [29].

### 2.6. qRT-PCR

Total RNA was extracted using TRIzol (Invitrogen, Carlsbad, CA, USA). RNA was reverse-transcribed into cDNA by a transcription kit (Takara, Dalian, China), and mRNA levels were measured via quantitative real-time PCR (qRT-PCR) [30]. The reactions were carried out using SYBR Premix Ex Taq™ (TaKaRa, Dalian, China). GAPDH was used as an endogenous reference [31]. The relative gene expression was evaluated by the 2^-*∆∆*CT^ method; each sample was measured at least three times.

### 2.7. Cell Transfection

LATS2 shRNA adenovirus and corresponding negative control (NC) were purchased from Guangzhou RiboBio Co., Ltd. (Guangzhou, China) and transfected into H9C2 cardiomyocytes by Lipofectamine™ 2000 (Invitrogen, CA, USA) [32, 33]. Cells were then incubated at 37°C in a humidified atmosphere with 5% CO_2_ for 6 h, and after another 48 h, they were collected for mRNA or protein analysis [34].

### 2.8. Statistical Analysis

The SPSS 18.0 software (SPSS Inc., Chicago, IL, USA) was used for data statistical analysis; the figures were plotted using GraphPad Prism (GraphPad, San Diego, CA, USA). Data were expressed as mean ± standard deviation (SD) [35]. The difference between groups was compared by Student's *t*-test or *χ*^2^ test.

## 3. Results

### 3.1. LATS2 Suppression Attenuates Hypoxia-Reoxygenation- (H/R-) Induced Cardiomyocyte Death

To determine the role of LATS2 in MIRI, we first analyzed the LATS2 expression in an in vitro hypoxia-reoxygenation (H/R) model in H9C2 cardiomyocytes. As shown in Figures 1(a) and 1(b), compared to the control group, the protein expression of LATS2 was rapidly upregulated after cardiomyocyte H/R injury. To analyze whether the increased LATS2 expression mediates the H/R-induced cardiomyocyte damage, we measured cell viability in H9C2 cardiomyocytes transfected with LATS2-adenovirus shRNA. As shown in Figure 1(c), control adenovirus shRNA transfection had no influence on cell viability. However, LATS2 shRNA transfection significantly increased cell viability after the H/R challenge, suggesting that LATS2 suppression is cardioprotective. To confirm these results, we analyzed apoptosis using the caspase-3/9 activity ELISA assay. As shown in Figures 1(d) and 1(e), compared to control, H/R treatment significantly elevated the caspase-3/9 activity, whereas transfection with LATS2 adenovirus shRNA reduced the caspase-3/9 activity. In addition, the LDH release cytotoxicity assay showed that the cardiomyocyte death induced by H/R injury could be attenuated by LATS2 knockout (Figure 1(f)). These results demonstrate that the H/R-induced cardiomyocyte death is mediated by LATS2.

### 3.2. LATS2 Suppression Improves Mitochondrial Function

Several molecular mechanisms have been proposed to explain the cardiomyocyte death in response to H/R injury [36–38]. Since a recent study suggested a relationship between LATS2 and mitochondrial dysfunction, we analyzed whether LATS2 decreases cardiomyocyte viability through inducing mitochondrial dysfunction. Mitochondrial damage is characterized by a reduced mitochondrial membrane potential [39]. Through immunofluorescence assay using the JC-1 probe, we observed a reduced mitochondrial membrane potential in cardiomyocytes after H/R injury (Figures 2(a) and 2(b)). Importantly, LATS2 suppression stabilized the mitochondrial membrane potential (Figures 2(a) and 2(b)). A reduced mitochondrial membrane potential impairs the mitochondrial respiration rate. As illustrated in Figures 2(c) and 2(d), the ELISA assay showed a decrease in mitochondrial state 3 and state 4 respiration after H/R injury. However, in cardiomyocytes transfected with LATS2 shRNA, mitochondrial state 3 and state 4 respiration was rapidly improved (Figures 2(c) and 2(d)). Mitochondrial respiration generates ATP, which is consumed by cardiomyocyte metabolism. As shown in Figure 2(e), the intracellular ATP production was blunted by H/R injury, but this decrease was not seen in cardiomyocytes transfected with LATS2 shRNA. These data indicate that LATS2 promotes mitochondrial membrane potential reduction, mitochondrial respiration delay, and ATP undersupply.

### 3.3. LATS2 Represses Mitochondrial Biogenesis by Suppressing PGC1*α*

There are two different mechanisms that repair damaged mitochondria: mitophagy and mitochondrial biogenesis [40, 41]. Mitophagy reduces the number of mitochondria through mitochondrial degradation [42, 43]. In contrast, mitochondrial biogenesis increases the number of mitochondria by enhancing mitochondrial regeneration and replication. The role of LATS2 in mitophagy has been investigated [44], but the influence of LATS2 on mitochondrial biogenesis has not been explored. Thus, we analyzed the markers related to mitochondrial biogenesis in cardiomyocytes after H/R injury and LATS2 suppression. As shown in Figures 3(a) and 3(b), compared to control, the gene expression of Tfam and Nrf1 was significantly reduced in cardiomyocytes after H/R injury, but LATS2 suppression increased the mRNA levels of Tfam and Nrf1 in cardiomyocytes.

Mitochondrial biogenesis is under the control of peroxisome proliferator-activated receptor gamma coactivator 1-alpha (PGC1*α*) [45, 46]. Thus, we analyzed whether LATS2 regulates the mitochondrial biogenesis through PGC1*α*. As shown in Figures 3(c) and 3(e), compared to control, H/R injury decreased the protein PGC1*α* levels in cardiomyocytes, but LATS2 suppression increased the protein PGC1*α* expression to near-normal levels. To understand the role of PGC1*α* in regulating the LATS2-mediated mitochondrial biogenesis, we analyzed the mitochondrial biogenesis markers in cardiomyocytes treated with SR-18292, a PGC1*α* inhibitor. As shown in Figures 3(f) and 3(g), the expression of Tfam and Nrf1 was significantly downregulated in response to H/R injury. Although LATS2 deletion reversed the mRNA levels of Tfam and Nrf1, this effect was negated by SR-18292 (Figures 3(f) and 3(g)). These results indicate that LATS2 represses mitochondrial biogenesis in H/R-treated cardiomyocytes by suppressing PGC1*α*.

### 3.4. PGC1*α* Inhibition Abolishes the Protective Effects of LATS2 Suppression in Cardiomyocytes

To determine whether the cardiomyocyte protection induced by LATS2 suppression is dependent on PGC1*α*, we analyzed cardiomyocyte viability in LATS2-suppressed H9C2 cells after PGC1*α* inhibition. As shown in Figure 4(a), LATS2 suppression sustained cardiomyocyte viability after H/R injury, whereas this protective action was abolished by SR-18292. Moreover, both caspase-3 and caspase-9 activities were inhibited by LATS2 deletion in H9C2 cells, whereas PGC1*α* inhibition reduced the protective effects of LATS2 deletion (Figures 4(b) and 4(c)). In addition, the LDH cytotoxicity assay showed that the LATS2 suppression-mediated cardioprotection was attenuated by SR-18292 (Figure 4(d)). Together, these results indicate that PGC1*α* inhibition abolishes the protective effects of LATS2 suppression in cardiomyocytes.

### 3.5. PGC1*α* Inhibition Promotes Mitochondrial Damage in LATS2-Deleted Cardiomyocytes

To find out if PGC1*α* is involved in the mitochondrial protection mediated by LATS2 suppression, we analyzed mitochondrial membrane potential in LATS2-suppressed H9C2 cardiomyocytes treated with SR-18292. As shown in Figures 5(a) and 5(b), LATS2 suppression was able to maintain mitochondrial membrane potential in H9C2 cells under H/R injury, but this beneficial action was undetectable in cardiomyocytes treated with SR-18292. Due to the impaired mitochondrial membrane potential, the mitochondrial state 3/4 respiration was also blunted in cardiomyocytes treated with SR-18292, although LATS2 suppression could reverse the mitochondrial respiration (Figures 5(c) and 5(d)). Finally, the ATP production was maintained at the baseline levels in response to LATS2 suppression after H/R injury, but SR-18292 was able to suppress the ATP synthesis, resulting in decreased ATP levels in H9C2 cardiomyocytes after H/R injury (Figure 5(e)). Together, these results indicate that LATS2 suppression protects mitochondrial homeostasis, and this action is dependent on the activity of PGC1*α*.

## 4. Discussion

The known mechanisms of MIRI include oxygen radical generation, mitochondrial damage, endoplasmic reticulum stress, intracellular Ca^2+^ ([Ca^2+^]i) overload, and cell apoptosis. Among them, cardiomyocyte apoptosis is one of the most important pathways and manifestations of MIRI. During MIRI, [Ca^2+^]i overload, increased mitochondrial permeability, and excessive accumulation of reactive oxygen species (ROS) can induce cardiomyocyte apoptosis, thereby aggravating the ischemia/reperfusion injury [47–49]. Therefore, it is important to identify mechanisms that regulate oxidative stress, [Ca^2+^]i concentration, and mitochondrial functions. Our *in vitro* results indicate that LATS2 is a critical regulator of cardiac MIRI. Hypoxia-reoxygenation (H/R) significantly increases the LATS2 expression in cardiomyocytes, whereas suppression of LATS2 maintains the mitochondrial functions and promotes cardiomyocyte survival. These findings identify LATS2 as a potential target for new personalized therapies against cardiac MIRI.

During MIRI, several cardioprotective signaling pathways are activated, especially the reperfusion injury salvage kinase (RISK) signaling. Other protective signals include protein kinase B (PKB, also known as AKT) and phosphatidylinositol 3 kinase (PI3K). The PI3K/AKT/glycogen synthase kinase 3*β* (GSK3*β*) pathway is a signal transduction pathway that plays important biological functions in cellular activities, such as apoptosis, survival, and proliferation [50–52]. PI3K phosphorylates phosphoinositides to generate phosphatidylinositol triphosphate, leading to activation of AKT. Activated AKT can further phosphorylate GSK3*β*, leading to cardioprotection. Studies have found that drug pretreatment can activate the PI3K/AKT/GSK3*β* signaling pathway in cardiomyocytes *in vivo* and *in vitro*, which plays an important role in the protection against MIRI [53–55]. Furthermore, studies have found that ischemic preconditioning can reduce myocardial infarct size after ischemia/reperfusion in mice, and indicated the AKT involvement. Activated GSK3*β* can open mitochondrial permeability transition pore and promote cell apoptosis, while inactivated GSK3*β* can protect cardiomyocytes and mitochondria from damage [56, 57]. Interestingly, the downstream effector of the above cardioprotective signaling mechanisms is the mitochondrial biogenesis. Mitochondrial biogenesis is the regenerative process that promotes mitochondrial turnover. In the present study, we found that mitochondrial biogenesis was inhibited after H/R injury. However, LATS2 deletion was able to restore the mitochondrial biogenesis and mitochondrial functions. These results indicate that LATS2 inhibits mitochondrial biogenesis.

The predictor of cardiac pathological changes is the LDH, which is a stable cytosolic enzyme in cardiomyocytes. When the myocardial cell membrane is damaged, LDH is rapidly released from the cells in the culture medium. Therefore, LDH can be used as an indicator of cell damage caused by H/R [58, 59]. Our data showed that LATS2 suppression significantly reduced the LDH content in the medium and this effect was dependent on the PGC1*α*-associated mitochondrial biogenesis [60–62]. In addition, the MIRI process is an oxidative stress process, where a large number of ROS are generated through multiple pathways [41, 45, 63]. The generated ROS cause dysfunction of cardiomyocytes, resulting in intracellular protein denaturation and degradation, and disruption of the cytochrome oxidase system, leading to energy metabolism disorders. We found that mitochondrial respiration and mitochondrial ATP production were blunted by H/R injury but returned to near-normal levels by LATS2 deletion. Future studies should determine whether LATS2 deletion also regulates the oxidative stress.

Apoptosis is one of the major forms of cell death during MIRI. Apoptosis is controlled by Bax and Bcl-2, belonging to the Bcl-2 family [64, 65]. While Bcl-2 inhibits apoptosis, Bax promotes apoptosis. Recent studies have found that the regulation of apoptosis is dependent on the Bcl-2/Bax ratio; the lower the Bcl-2/Bax ratio, the more severe the apoptotic condition tends to be [66, 67]. The caspase protein family plays an important role in the initiation and regulation of apoptosis. Caspase-3 is a key caspase activated by various apoptotic stimuli [68, 69]. Our results showed that cardiomyocyte apoptosis could be attenuated by mitochondrial biogenesis in a manner dependent on LATS2 deletion, suggesting that LATS2 is a new regulator of cardiomyocyte apoptosis.

Together, our results demonstrate that mitochondrial damage is a primary feature of cardiomyocyte hypoxia-reoxygenation injury in vitro. LATS2 overexpression promotes cardiomyocyte death and mitochondrial damage through suppression of mitochondrial biogenesis. Therefore, approaches targeting LATS2 or mitochondrial biogenesis will be further tested in the clinical management of cardiac MIRI.

## Figures and Tables

**Figure 1:** LATS2 deletion attenuates hypoxia-reoxygenation- (H/R-) mediated cardiomyocyte death. (a, b) Western blot analysis of LATS2 in H9C2 cardiomyocytes. (c) Cell viability was measured by CCK-8 assay in H9C2 cardiomyocytes transfected with LATS2-adenovirus shRNA. (d, e) ELISA analysis of caspase-3/9 activity. (f) LDH release assay was used to analyze the cell viability. ^∗^*p* < 0.05.

**Figure 2:** LATS2 deletion improves mitochondrial function. (a, b) JC-1 assay was applied to analyze the changes in mitochondrial membrane potential. (c, d) ELISA was used to detect the changes in mitochondrial state 3 and state 4 respiration. (e) ATP production was determined through ELISA. ^∗^*p* < 0.05.

**Figure 3:** LATS2 represses mitochondrial biogenesis by downregulating PGC1*α*. (a, b) qRT-PCR analysis of Tfam and Nrf1 mRNA levels in cardiomyocytes. (c–e) Western blot analysis of PGC1*α* expression. (f, g) qRT-PCR analysis of Tfam and Nrf1 mRNA levels in H9C2 cardiomyocytes after treatment with SR-18292, a PGC1*α* inhibitor. ^∗^*p* < 0.05.

**Figure 4:** PGC1*α* inhibition abolishes the protective effects of LATS2 deletion in cardiomyocytes. (a) Cell viability was measured by CCK-8 assay in H9C2 cardiomyocytes transfected with LATS2-adenovirus shRNA and treated with SR-18292. (b, c) ELISA was used to analyze the activity of caspase-3. (d) LDH release assay was used to analyze the cell viability. ^∗^*p* < 0.05.

**Figure 5:** PGC1*α* inhibition promotes mitochondrial damage in LATS2-deleted cardiomyocytes. (a, b) JC-1 analysis of mitochondrial membrane potential. (c, d) ELISA was used to detect the changes in mitochondrial state 3 and state 4 respiration. (e) ATP production was determined through ELISA. ^∗^*p* < 0.05.

## Data Availability

The data of this study are available from the corresponding author upon request.
